This article has been retracted.

# The prognostic value of prognostic nutritional index in hepatocellular carcinoma patients: A meta-analysis of observational studies

**DOI:** 10.1371/journal.pone.0202987

**Published:** 2018-10-12

**Authors:** Zhiling Wang, Jie Wang, Peijun Wang

**Affiliations:** 1 Department of SICU. Affiliated Children 's Hospital of Zhengzhou University, Henan Children's Hospital, Zhengzhou, Henan Province, China; 2 General Surgery, Affiliated Tumor Hospital of Zhengzhou University, Henan Provincial Cancer Hospital, Zhengzhou, Henan Province, China; Universita degli Studi di Pisa, ITALY

## Abstract

**Background and aims:**

The clinical value of the prognostic nutritional index (PNI) in hepatocellular carcinoma (HCC) has been investigated in previous studies, but the results remain controversial. Here we present a meta-analysis to systematically review the association between PNI and HCC prognosis.

**Method:**

PubMed, EMBASE, Web of Science databases were systematically searched to identify relevant studies. Data were abstracted independently by two reviewers. A meta-analysis was performed to determine the prognostic and clinic-pathological values of PNI in HCC patients. Odds ratios (ORs) and 95% confidence intervals (CIs) were extracted to estimate the association of PNI with survival and clinic-pathological characteristics, respectively.

**Results:**

A total of eleven studies involving 3165 patients were analyzed. The pooled results indicated that low PNI is a significant predictor of poor 1-year, 3-year, 5-year OS (OR, 2.91, 4.05, 3.65; 95%CI, 2.30 to 3.70, 3.27 to 5.03,2.96–4.50; P = 0.14,0.22,0.11 respectively) and disease-free survival (DFS) (OR,2.35, 2.57, 2.75; 95%CI, 1.71 to 3.23, 1.89 to 3.49,2.01 to 3.75; P = 0.39,0.04,0.11, respectively). Moreover, PNI is significantly associated with serum AFP, tumor recurrence, tumor size and TNM stages in HCC patients. However, PNI is not significantly associated with tumor number and the incidence of cirrhosis in HCC patients.

**Conclusions:**

PNI is an independent predictive indicator of survival and associated with serum AFP, tumor recurrence, tumor size and TNM stages in HCC patients.

## Introduction

Hepatocellular carcinoma (HCC) is one of the most common malignancies [1], the third leading cause of cancer-related death in the word [2], Unlike other solid malignancies, most hepatocellular carcinoma evolved from chronic liver disease, especially associated with liver cirrhosis result from viral hepatitis or ethanol consumption [3,4]. Despite remarkable development in early diagnosis, surgery, adjuvant chemotherapy, even liver transplantation, but the effect remains unsatisfactory because of the high recurrence rate or metastasis within 5 years after treatment in HCC patients [5]. Therefore, it is important to assess disease progression in a timely manner and guide clinical treatment to improve the survival of patients.

Immune-nutritional status has been demonstrated to be associated with prognosis in patients with various malignancies and inflammatory response was known to promote tumor growth, invasion, angiogenesis and metastasis [6–8]. Prognostic nutritional index (PNI) based on albumin concentration and lymphocyte count in the peripheral blood, is a simple and practical indicator of systemic inflammatory response [9]. Recently, emerging evidence has reported the prognostic value of PNI in hepatocellular carcinoma [10–12]. However, those studies that using the PNI for HCC prognosis reported inconsistent results, largely due to differences in inclusion criteria and sample sizes [13, 14], as a result, the correlation of PNI with survival in HCC patients remains controversial. The aim of this study is to perform a meta-analysis to determine whether PNI is a useful prognostic factor and assess the correlation between PNI and clinic-pathological parameters in HCC patients.

## Materials and methods

### Search strategy

PubMed; EMBASE and Web of Science databases were comprehensively searched for relevant studies published from 1980 to December 2017 with the following keywords: “hepatocellular carcinoma”, “hepatocellular tumor”, “hepatocellular malignance” and “Prognostic nutritional index”, “PNI” and“prognosis”, “survival”, “outcome”. No time and language restrictions were imposed. Additionally, the relevant literatures including all of the identified studies, reviews and editorials were also reviewed. All candidate studies were carried out by two independent reviewers (Zhiling Wang and Peijun Wang) and discrepancies were resolved by consensus.

#### Criteria for inclusion and exclusion

Studies that fulfilled the following criteria were considered eligible and selected into this article: (1) pathologic examination for diagnosis of hepatocellular carcinoma; (2) clinic-pathological and prognostic values of PNI in HCC was reported; (3) case-control studies design; (4) sufficient data to allow for estimation of the OS, DFS. Nonhuman hepatocellular carcinoma research studies, duplicate articles, abstracts, recurrent HCC, letters, case reports and meetings reports were excluded from the analysis. Two reviewers evaluated all candidate literature and resolved any disagreement by discussion.

#### Data extraction

Two independent investigators reviewed the publications and extracted the data from relevant identified: author’s first name, year of publication, country, sample size, TNM stages, follow-up period, cutoff value and outcomes.

#### Quality assessment

In the included studies, PNI was calculated on the basis of pretreatment laboratory data and was using the formula: 10×albumin value (g/dl) + 0.005×lymphocyte count in the peripheral blood. The quality of the included studies was assessed using the Newcastle-Ottawa quality assessment scale (NOS) and we considered studies awarded with 6 or higher were classified as high-quality studies [15].

### Statistical analysis

Meta-analysis was conducted using Review Manager 5.3 analysis software (Cochrane Collaboration, Copenhagen, Denmark). The association of PNI with survival and clinic-pathological characteristics in HCC patients were performed using ORs and 95% CI. The estimates of ORs were weighted and pooled using the Mantel-Haenszel fixed effects model. Statistical heterogeneity was assessed using the Cochran’s Q and I2 statistics, if I2 ≥ 50% or/and P < 0.10 were used to indicate statistically significant heterogeneity and a random-effects model was applied. Otherwise, a fixed-effect model was used [16]. Publication bias was assessed by visual inspection of the funnel plot. All statistical tests were two-sided, and statistical significance was defined as *P<*0.05.

## Results

### Eligible studies

A total of 39 potentially relevant studies were retrieved from three databases by the initial search.

A flow chart showing the study selection was presented in S1 Fig. The initial search identified 39 studies, of which eleven studies by comprising 3165 patients published from 2012 to 2017 were finally included in this meta-analysis [17–27]. Eight studies from China, Two studies from Japan and one from UK. Study characteristics are presented in S1 Table.

### PNI and Overall survival (OS) in HCC

There eleven studies reported the prognostic value of PNI for OS. Eleven studies reported the 1-year OS, ten studies and eight studies described the 3-year OS, 5-year OS, respectively. The results indicated that low PNI is significantly associated with poor prognosis of 1-year, 3-year and 5-year OS, without heterogeneity (OR, 2.91, 4.05, 3.65; 95%CI, 2.30 to 3.70, 3.27 to 5.03, 2.96–4.50; I^2^ = 33%, 24%, 0%; P = 0.14, 0.22, 0.11 respectively), these results suggested that low PNI predict a poor OS in HCC patients. (S2 Fig)

### PNI and disease-free survival (DFS) in HCC

DFS was mentioned in four studies. The pooled estimate for DFS indicated low PNI is significantly associated with poor prognosis of 1-year, 3-year and 5-year DFS in HCC patients (S3 Fig). A random-effects model was applied to calculate the pooled OR and 95%CI because of significant heterogeneity (OR, 2.35, 2.57, 2.75; 95%CI, 1.71 to 3.23, 1.89 to 3.49, 2.01 to 3.75; I^2^ = 0%, 68%, 55%; P = 0.39, 0.04, 0.11 respectively). The results indicating that low PNI is likely to predict shorter DFS.

### Relationship between PNI and clinic-pathological features

#### PNI and tumor stage

Four studies presented the data that about PNI and tumor stage in HCC patients. Our results indicated that low PNI have lower incidence of I and II stage (OR = 1.9, 95% CI = 1.22–1.96, P < 0.01), but there have no statistically significance in the stage III and IV between high PNI group and low PNI group (OR = 0.74, 95% CI = 0.55–1.01, P = 0.06) (S4A Fig).

#### PNI and cirrhosis

Five studies reported the association between PNI and the incidence of cirrhosis, the pooled results indicated that PNI have no significant association with the incidence of cirrhosis (OR = 0.86, 95% CI = 0.65–1.12, P = 0.26) (S4B Fig).

#### PNI and tumor number

Six studies reported tumor number (single or multiple), the pooled results suggested that PNI have no correlation with tumor number in HCC patients (OR = 0.89, 95% CI = 0.45–1.75, P = 0.11) (S4C Fig).

#### PNI and tumor size

Tumor size(≥5cm or <5cm)was reported in 4 studies, the pooled result indicated that low PNI group have a higher incidence of large tumor (OR = 0.52, 95% CI = 0.40–0.67, P = 0.004)(S5A Fig).

#### PNI and AFP

Five studies provided data about the correlation between PNI and serum AFP, the pooled results suggested that low PNI group have a higher serum AFP than high PNI group (OR = 0.51, 95% CI = 0.32–0.8, P = 0.003)(S5B Fig).

#### PNI and tumor recurrence

Tumor recurrence was reported in four studies, the pooled results suggested that low PNI have a higher recurrence incidences (OR, 0.37; 95% CI 0.23 to 0.59; I2 = 47%; P<0.01) (S5C Fig).

### Publication bias

A funnel plot was used to assess the included studies for overt publication bias showed symmetry for OS and DFS (S6 Fig).

## Discussion

Some studies reported that the prognosis of hepatocellular carcinoma patients have a close relation with tumor burden, liver function and body immune status [28, 29]. Currently, recurrence and metastasis of hepatocellular carcinoma is still the most important reason for treatment failure. There are some factors that lead to recurrence include tumor size, vascular invasion, liver function, cirrhosis, immune status and so on. To our knowledge, the prognostic and clinic-pathological value of PNI has recently been studied in patients with many malignancies. However, the prognostic and clinic-pathological role of PNI in HCC patients is still not reported. This is the first systematic review/meta-analysis to provide a prognostic role of PNI and the relationship between PNI clinic-pathological characteristics in patients with HCC.

Eleven non-randomized trials compared the prognostic effects of PNI in HCC patients. Our results indicated that low PNI is a poor prognostic factor for OS and DFS in patients with HCC. These pooled results suggested that high PNI is a beneficial to the survival of HCC patients and associated with more favorable outcomes such as lower AFP, lower recurrence, minor tumor size and better TNM. However, PNI does not compromise clinic-pathological features including tumor number and the incidence of cirrhosis. Given these data, a simple PNI was shown to be a promising predictor of survival in HCC patients.

Several potential mechanisms may reveal that why low PNI is associated with poor prognosis in HCC patients. First, more and more evidences confirm that systemic inflammatory response plays a significant role in the development and progression of HCC. PNI which is a combination of the albumin and total lymphocyte count, was initially used to evaluate the immunological and nutritional aspects of patients undergoing surgery of the gastrointestinal tract [30]. Low PNI may be the result of hypoalbuminemia and/or lymphocytopenia. Albumin as the main component of plasma proteins, hypoalbuminemia reflected the presence of cancer cachexia is caused by a sustained inflammatory response, either from the tumor itself or as a host reaction [31]. However, impaired synthetic functions accompanying cirrhosis needs to be considered as an additional determinant of reduced serum albumin. Lymphocytes are crucial components of the immune system, play an extremely important role in the biological behavior of HCC, such as initiation, proliferation, differentiation and metastasis [32, 33], affect the tumor microenvironment, prevent tumorigenesis and recurrence by generating cytokines and causing the cytotoxic effect of cancer cell death [34], so antitumor effect induced by the cellular immunity of T lymphocytes decreased because of lymphocytopenia [35]. Therefore, PNI reflects both the nutritional and immunological status of the host and can be a predictor of prognosis in HCC patients. Indeed, our findings indicated that PNI was an independent prognostic factor on OS and DFS in HCC patients and consistent with the above evidences. Second, our results indicated that low PNI was associated with more advanced tumor features, such as tumor recurrence, tumor size, serum AFP and TNM. The present meta-analysis showed that PNI was related to tumor recurrence and TNM, which might be explained by the immunological status. However, the correlation between PNI and serum AFP worth further study.

The synthesis of albumin is involved in HCC patients accompanied with cirrhosis [36], so we studied the correlation between PNI and the incidence of cirrhosis, the pooled results indicated that there is no obvious correlation between PNI and the incidence of cirrhosis. Mengyun Ke et al found that PNI was associated with tumor number in HCC patients [37], we analyzed the six studies included in this meta-analysis, pooled results suggested that PNI have no correlation with tumor number in HCC patients.

There were several limitations in our meta-analysis. First, all the included studies were retrospective cohort studies. Second, we could not perform other subgroup analyses because of the limited number of studies included. Third, those studies included in this meta-analysis mainly from Asian countries, only one from Europe.

### Conclusion

In summary, our study suggests that PNI may be a potential marker to predict the prognosis of HCC patients.

## Supporting information

S1 Checklist PRISMA checklist. (DOC)

S1 Table Characteristics of the included studies. (TIF)

S1 Fig Flow chart of literature search and study selection. (TIF)

S2 Fig Forest plots depicting 1-year OS, 3-year OS and 5-year OS reported in the included studies. ORs are shown with 95% CIs. CI: confidence interval.
(TIF)

S3 Fig Forest plots depicting 1-year DFS, 3-year DFS and 5-year DFS reported in the included studies. (TIF)

S4 Fig Forest plots depicting tumor TNM (A), the incidence of cirrhosis (B) and tumor number(C).
(TIF)

S5 Fig Forest plots depicting tumor size (A), serum AFP (B) and the incidence of recurrence(C).
(TIF)

S6 Fig Begg’s Funnel plot for evaluation of publication bias in OS and DFS. (TIF)
